# Mechanism of action of novel piperazine containing a toxicant against human liver cancer cells

**DOI:** 10.7717/peerj.1588

**Published:** 2016-03-17

**Authors:** Nima Samie, Sekaran Muniandy, MS Kanthimathi, Batoul Sadat Haerian

**Affiliations:** 1 Department of Pharmacology, Faculty of Medicine, University of Malaya, Kuala Lumpur, Malaysia; 2 Department of Molecular Medicine, Faculty of Medicine, University of Malaya, Kuala Lumpur, Malaysia; 3 University of Malaya Centre for Proteomics Research, Faculty of Medicine, University of Malaya, Kuala Lumpur, Malaysia

**Keywords:** Cytoskeletal rearrangement, Piperazine, Apoptosis, Liver cancer

## Abstract

The purpose of this study was to assess the cytotoxic potential of a novel piperazine derivative (PCC) against human liver cancer cells. SNU-475 and 423 human liver cancer cell lines were used to determine the IC50 of PCC using the standard MTT assay. PCC displayed a strong suppressive effect on liver cancer cells with an IC50 value of 6.98 ± 0.11 µM and 7.76 ± 0.45 µM against SNU-475 and SNU-423 respectively after 24 h of treatment. Significant dipping in the mitochondrial membrane potential and elevation in the released of cytochrome c from the mitochondria indicated the induction of the intrinsic apoptosis pathway by PCC. Activation of this pathway was further evidenced by significant activation of caspase 3/7 and 9. PCC was also shown to activate the extrinsic pathways of apoptosis via activation of caspase-8 which is linked to the suppression of NF-*κ*B translocation to the nucleus. Cell cycle arrest in the G1 phase was confirmed by flow cytometry and up-regulation of glutathione reductase expression was quantified by qPCR. Results of this study suggest that PCC is a potent anti-cancer agent inducing both intrinsic and extrinsic pathways of apoptosis in liver cancer cell lines.

## Introduction

Liver cancer is the sixth most frequent cause of cancer deaths worldwide and hepatocellular carcinoma is the most common form of liver cancer in adults (Siegel, Miller & Jemal, 2015). Cancer is initiated by turning normal cells into tumors through environmental factors such as carcinogens, viruses, chemicals, and radiation as well as by genetic conditions such as germline mutations leading to malignant growth, and invasion and metastasis. Despite the significant progress in diagnosis of liver cancer and using a combination of different modalities, including surgery, chemotherapy, and radiotherapy, the remission, relapse, and metastasis are still more frequent than other cancers and the five-year relative survival rate is approximately only 15% (Ferlay et al. (2012)). Failure of programmed cell death is a key contributor to both development of cancer and responsiveness to drugs (Brown & Attardi, 2005). Apoptotic pathways are regulated by a number of gene families which finally lead to the phagocytosis of cells by adjacent cells. Extrinsic and mitochondrial (intrinsic) pathways are considered as main controllers of apoptosis (Thangam et al., 2014). Although chemotherapy-induced apoptosis is the main approach of numerous anti-cancer therapies, several drugs have been implicated in the emergence of treatment resistance and side effects (Kranz & Dobbelstein, 2012). Discovery of potent drugs targeting apoptosis signal transduction are warranted to ameliorate clinical consequences in cancer therapy (Ahmed & Van Etten, 2013). Piperazines are nitrogen containing heterocyclic compounds and constitute the functional group in several drug backbones which enable them to display a broad range of biological activities such as oxidation and anti-inflammation (Asif, 2015; Siddiqui et al., 2011). These agents possess a flexible binding feature with a general binding motif which offers potent and selective ligands for a variety of biological targets (Berkheij et al., 2005). Furthermore, interaction with DNA is another outstanding feature of a compound containing piperazine substituents (Wilson et al., 1990). On the basis of these properties, piperazines have been used as anticancer (Gillet et al., 1997; Hulme & Cherrier, 1999), antifungal (Upadhayaya et al., 2004), antibacterial and antimalarial agents (Chaudhary et al., 2006). Effective anti-proliferative activity against colon and breast cancer and leukemia has been exhibited by piperazine analogues (Yoshida, Maehara & Sugimachi, 1999). Piperazine containing compounds are more potent and active than the taxane family, sorafenib, cisplatin and doxorubicin in recent studies, and are widely prescribed chemotherapeutic drugs against different tumors (Hatnapure et al., 2012). Direct induction of apoptosis is a prominent trait of piperazines in the destruction of tumor cells, suggesting this compound as an anticancer drug candidate. The aim of this study is to evaluate the cytotoxic properties of (2, 4-Dihydroxy-cyclohexyl)-[4-(3, 5-dihydroxy-cyclohexyl)-piperazin-1-yl]-methanone designated as PCC against human liver cancer cells. We determined the potency of PCC in the induction of apoptosis.

## Material and Methods

### Purification procedure

The spectrophotometric analysis for PCC in hydrochloric acid (0.01 mole/l) was performed using a UV/VIS Lambda 20 (Perkin Elmer) spectrophotometer. The specific absorption coefficient and the molar absorbancy index for PCC were calculated based on the Lambert–Beer equation. The solutions of PCC were prepared over a concentration range from 0.00098% to 0.00141%. The course of hydrolysis in an acidic medium (at HCl 0.1 mole/l, pH = 1.11 and 60 °C) was followed by the TLC method using plastic sheets 20 × 20 cm with silica gel (0.2 mm) 60 F 254 (Merck). A thin-layer chromatographic tank with a flat bottom of trans-parent glass of size 27.5 × 27.5 × 7.5 cm was suitable. The chromatographic solvent consisted of a mixture of butanol-acetic acid (1.05 kg/l)—water (80: 12: 30). The solvent system advanced approximately 15 cm in about 6 h. Visualization-UV light 254 and 365 nm (ENF-260C/F; Spectroline, New York, USA) and ninhydrine reagent. Decomposition of PCC was observed using the HPLC method. The analytical system consisted of a Rheodyne 7120 20 ml fixed-loop injector, an LC 3-UV detector (Pye Unicam, England), an L-6000 A pump (Merck- Hitachi, Germany) and an A/C transmitter with the software Chromed (Medson, Poland). An LiChrosorb 100 RP-18 column 250 × 4.0 mm I. D., *dp* = 5 µm (Merck) was used. The mobile phase consisted of acetonitrile and phosphate buffer (0.01 mole/l, pH = 2) (50: 50-phase A) or (30: 70-phase B). The flow rate was 1.5 ml/min. UV detection was carried out at 239 nm. The final concentration of internal standard solution was 50 mg/ml. To validate the HPLC method, the solutions of PCC in HCl (0.01 mole/l) were used as the solution of analyte. The precision of the method was determined through the analysis of 6 replicate injections of standard solution containing 25.0, 50.0 and 75.0 mg/ml of substance PCC dissolved in HCl (0.01 mole/l). The linearity between *p*∕*pi* (*p*, *pi*-areas of substance PCC and internal standard concentrations of PCC in HCl (0.01 mole/l) ranging from 5.1 mg/ml to 204.0 mg/ml was examined for 10 points of 3 replicate injections. For kinetical interpretation of hydrolysis, the solutions of PCC (0.430 mg/ml) in HCl (0.1 mole/l, pH = 1.11, *m* = 0.50 mole/l) or in NaOH (0.1 mole/l, pH = 13.06, *m* = 0.50 mole/l) were stored at 60 °C or 37 °C and concentration changes of substance PCC in the course of time were recorded. To each 1.0 mL sample to be analysed, 1.0 mL of internal standard (0.15 mg/mL) and 1.0 ml of water were added. PCC molecular mass was found −394.47; elementary composition: 66.99 (66.88) %C, 6.64 (6.82) %H, 14.20 (14.38) %N; melting point 131 °C–133 °C.

### Cell culture

Human liver cell line (THLE-3) and cancer cell lines (SNU-475 and SNU-423) were purchased from American Type Culture Collection (ATCC, Manassas, Virginia, USA). SNU-475 and 423 were cultured in Roswell Park Memorial Institute medium (RPMI-1640) supplemented with 10% heat inactivated fetal bovine serum (FBS; Sigma-Aldrich, St. Louis, MO) and 1% penicillin and streptomycin. THLE-3 was grown in Bronchial Epithelial Cell Growth Medium (BGEM) bulletkitTM (Lonza/Clonetics Corporation, Walksrsville, MD 21793). All cell lines were cultured in a humidified incubator with 5% CO_2_ at 37 °C. All experiments were conducted on cell lines with passage number 1–10.

### Cell viability assay

The MTT [3-(4, 5-Dimethylthiazol-2-yl)-2, 5-Diphenyltetrazolium Bromide] assay was carried out to evaluate the anti-proliferative activity of PCC. Briefly, cells were seeded 24 h prior to treatment in a 96-well plate at 7 × 10^4^ cells/ml. PCC and 5-fluoruracil (standard) were dissolved in DMSO (Sigma Chemical Co., St. Louis, Missouri, USA). After incubation of the plate for 24, 48 and 72 h at 37 °C with 5% CO_2_, 50 µl of MTT solution (2 mg/ml; Sigma) was added to each well. The plates were then incubated for 24 h under the same conditions. To dissolve the purple formazan crystals formed at the bottom of the wells, 200 µl DMSO was added to each well and incubated for 20 min. Absorbance was subsequently read at 570 nm using a spectrophotometric plate reader (Hidex, Turku, Finland). Experimental data were derived from three independent experiments. The selectivity index was obtained by mean IC50 THLE-3/mean IC50 of SNU-475 or SNU-423.

### Immunofluorescence

After 24 h PCC treatment of both cancer and normal cells, 10 µg/ml JC-1 mitochondrial membrane potential dye (eBioscience, San Diego, CA) were added to the live cells followed by incubation for 30 min at 37 °C. Cells were then fixed in 4% paraformaldehyde, permeabilized by 0.25% Triton X-100, quenched with 50 mM ammonium chloride and blocked with 5% BSA in PBS overnight, followed by probing with 5 µg/mL anti-cytochrome c antibody (Alexa Fluor 488; Abcam Inc., Cambridge, MA, USA) for 1 h. 10 µg/mL DY350-Phalloidin and 4 µg/mL Hoechst 33342 (Thermo Scientific, Hudson, NH, USA) were added into the staining solution and cells were incubated at room temperature for 20 min. Finally, cells were washed with PBS and coverslips were mounted using polyvinyl alcohol mounting medium (Fluka Analytical, Milan, Italy). Fluorescence was analysed using the Radiance 2100 confocal microscope (Bio-Rad, Hercules, CA, USA). Noise reduction was attained by Kalman filtering during application and data were analyzed with Data Viewer version 3.0.

### Cell cycle analysis using flow cytometery

Briefly, cells were treated with PCC (6.25 µg/ml) for 24 h. DMSO was served as negative control. BrdU and Phospho-Histone H3 dyes were added to the treated cells for 30 min. After fixation, the cells were observed and analysed using a Cellomics Array Scan HCS reader (Thermo Scientific). Following incubation of the cells with PCC (6.25 µg/ml) for 24, 48 and 72 h, cells were centrifuged at 1,800 rpm for 5 min and followed by mixing the cell pellets with 700 ml of cold 90% ethanol and mentioned at 4 °C overnight. Cells were washed and suspended in PBS and 25 ml RNase A. 50 ml of propidium iodine was then added to the fixed cells followed by incubation for 1 h at 37 °C. The DNA content of the cells was analysed using CytoFLEX Flow Cytometer (Beckman Coulter Inc., CA, USA).

### Live/dead cell determination

Accurate determination of live/dead nucleated cell concentration in the sample was accomplished by the minor modified version of the method described by Rahman et al. (2014). Propidium iodide (PI) and acridine orange (AO) double staining assay was performed to detect the early and late apoptotic properties of the treated cancer cells according to the standard procedure. Cells were incubated with PCC (6.25 µg/ml) for 24, 48, 72 h and the harvested cells were stained with acridine orange and propidium iodine and observed within 30 min using a UV-fluorescent microscope (Bio-Rad, Hercules, CA, USA).

### Quality assay of apoptosis

Cells were treated with cell membrane permeable calcium chelator (EGTA/AM, 25 µM; Life Technologies, Gaithersburg, MD, USA) for a period of 1 h prior to addition of PCC (6.25 µg/ml). After 24 h treatment, cells were harvested, washed twice with PBS, resuspended in Annexin-V binding buffer (BD Biosciences, San Jose, CA, USA) and stained with Annexin-V-FITC (BD) and PI (sigma) according to the manufacturer’s protocol. The fluorescence intensity was then examined using CytoFLEX Flow Cytometer (Beckman Coulter Inc., CA, USA). Annexin-V was used for determination of early and late apoptosis, whereas PI was used for distinguishing necrosis and late apoptosis.

### Determination of antioxidant potential

Organisms have complex antioxidant systems to protect themselves from oxidative stress; however, excessive oxidative stress can overwhelm the system and cause severe damage. To measure the antioxidant protection potential of PCC over time, the oxygen radical absorbance capacity (ORAC) assay was used. In a black 96-well plate, 6.25 µg/ml of PCC, blank (solvent/PBS) and standard (5-fluouracil) were added to cells supplemented with fluorescein solution (150 µl) and incubated at 37 °C for 5 min. AAPH (25 µl) was then added and fluorescence intensity was assessed at 485 nm (excitation wavelength) and 538 nm (emission wavelength) every 2 min for duration of 2 h. Quantification was carried out by calculating the differences of area under the fluorescence decay curve of the samples and blank.

### Detection of ROS production

ROS is produced as byproducts during mitochondrial electron transport and has potential to cause apoptosis. Intracellular reactive oxygen species were measured by using 10 mM dihydroethidium (DHE) stock solution (in methanol) diluted 500-fold in HBSS without serum or other additives to yield a 20 mM working solution. The cells in the black plate were washed twice with HBSS after exposure to PCC following incubation of 100 ml DHE working solution at 37 °C for 30 min. Fluorescence intensity of DCF was analyzed using Radiance 2100 confocal microscope (Bio-Rad, Hercules, CA, USA).

### LDH release analysis

Quantitative measurement of lactate dehydrogenase (LDH) released into the media from damaged cells as a biomarker for cellular cytotoxicity and cytolysis was carried out according to Wang, Grunz-Borgmann & Parrish (2014) with slight modifications. Briefly, cells were treated with different concentrations of compound PCC and Triton X- 100 (positive control) for 48 h followed by transfer of the supernatants of untreated and treated cells to a new 96-well plate for LDH activity analysis. 100 µL of LDH reaction solution was then added to each well, followed by incubation at room temperature for 30 min. The absorbance was read at 490 nm using a Tecan Infinite 200 Pro (Tecan, Mannedorf, Switzerland) microplate reader. LDH activity of the cells was assessed by the amount of formazan salt and intensity of red color in treated and untreated samples. Release of LDH level in treated cells was expressed as a percentage of LDH release in the positive control.

### Evaluation of NF-*κ*B translocation

Nuclear factor kappa-light-chain-enhancer of activated B cells controls transcription of DNA and is involved in cellular responses to stimuli such as stress, free radicals and chemicals. Cells were treated with (6.25 µg/ml) and stimulated with TNF-*α*. The Cellomics nuclear factor-*κ*B (NF-*κ*B) activation kit (Thermo Scientific) was used for staining of the cells. The average intensity ratio (200 cells/well) of the nuclear and cytoplasmic NF-*κ*B was measured using cytoplasm to nucleus translocation bio-application software (S50-5001-1, Thermo Scientific).

### Evaluation of gene expression in the cells

SNU-475 and SNU-423 cells were treated with PCC (6.25 µg/ml) for 24 h. Total RNA was extracted using RNeasy plus mini kit (Qiagen). Reverse transcription of 1 mg RNA into cDNA was carried out by using RT2 first strand kit (SA Biosciences, Qiagen). TR2 Real Time TM SYBR Green/fluorescein PCR master-mix was then mixed with cDNA and loaded into each of the 96 wells of the 84 genes by qPCR array according to the manufacturer’s protocol (SA Biosciences, Qiagen). Differential expression of the members of antioxidant peroxiredoxin (PRDX) family and redox control which are involved in human oxidative and cellular stress were analyzed. Concisely, 12.5 ml master mix, 11.5 ml double distilled water, and 1 ml cDNA was mixed to a final volume of 25 ml PCR mixture and loaded into each well of the 96-well plate. QuantStudio™ 12 K Flex Real-Time PCR system consuming ssoFast EvaGreen Supermix (Bio-Rad) was carried out according to the manufacturer’s protocols. Primes were synthesized as GR F5′-AACATCCCAACTGTGGTCTTCAGC-3′, GR R5′ TTGGTAACTGCGTGATACATCGGG-3′, ß-actin F5′-GATGACCCAGATCATGTTT GAGACC-3′ and ß-actin R5′ AGTCCATCACGATGCCAGTGGT-3′. Amplification was operated at 95 °C for 10 min, followed by 40 cycles at 95 °C for 15 s and 60 °C for 1 min. The average expression of five housekeeping genes including *β*-actin (ACTB), *β*-2-microglobulin (B2M), hypoxanthine phoshoribosyltransferase 1 (HPRT1), ribosomal protein L13 a (RPL13A) glyceraldehyde-3-phosphate dehydrogenase (GAPDH) was considered for normalization of mRNA expression of each gene. The difference in gene expression between piperazine and untreated control was calculated by RT Profiler qPCR-array data analysis software to measure the fold changes.

### Evaluation of mitochondrial and extrinsic apoptotic pathways

Caspases are a family of cysteine proteases that have critical roles in apoptosis. Caspase 9 is involved in the intrinsic, whereas. Caspase 8 is involved in the extrinsic pathway of apoptosis. Caspase 3 interacts with caspase 8 and 9 and plays a central role in the execution-phase of the cell apoptosis. Time-dependent evaluation of caspase 3/7, 8 and 9 activities in the presence of PCC (6.25 µg/ml) were performed using assay kits, Caspase-Glo 3/7, 8 and 9 (Promega Corp., Madison, WI, USA) in triplicates on white 96-well plates after 6, 12, 18, 24 and 30 h. Treatment with PCC (6.25 µg/ml) was carried out on a total of 10,000 cells per well and 100 ml of the Caspase-Glo reagent added and incubated at room temperature for 30 min. Cleavage of the aminoluciferin-labeled synthetic tetrapeptide based on the caspase activation, causes apoptotic cells to release the substrate of luciferase enzyme. Activity of caspase was evaluated using Tecan Infinite 200 Pro (Tecan, Mannedorf, Switzerland) microplate reader.

### Molecular identification of apoptotic proteins induced by PCC

Apoptotic proteins have a central role in regulation of programmed cell death via inducing (pro-apoptotic) or inhibiting (anti-apoptotic) apoptosis. 1 × 10^6^ cells/ml were treated with PCC and standard (5-fluorouracil) separately for 24 h. Cells were then aspirated, lysed and resolved on 10% SDS-polyacrylamide gels followed by transferring of the proteins to PVDF membranes (Milipore) and blocking with 5% nonfat dry milk in PBS-T (0.05% Tween 20) for 1 h at room temperature. Primary antibodies, included Bid(1:1000), caspase-3 (1:1000), caspase-8 (1:1000), caspase-9 (1:1000), anti *β*-actin (1:5000), Bax (1:1000) Santa Cruz Biotechnology Inc. (Santa Cruz, CA, USA), Bcl-xL (1:1000), Bcl-2 (1:1000), p53 (:1000) (Abcam Inc., Cambridge. MA, USA). Secondary antibodies conjugated to horseradish peroxidase were obtained from Kirkegaard & Perry Laboratories Inc. (Gaithersburg, MD, USA). Protein-antibody complexes were detected using Amersham ECL prime Western blotting detection reagent (GE Healthcare, Munich, Germany).

### Statistical analysis

All values are expressed as mean ± S.D. Student’s *t*-test was used for statistical evaluation of data. A probability value of ^∗^*p* < 0.05 was considered statistically significant.

## Results

### Purification grade of PCC

The TLC-system ensured a chromatographic separation of PCC following hydrolysis in HCl. The limit of detection (LOD) for PCC was found to be 1 µg for detection in UV-light at 254 nm. A mixture of acetonitrile in phosphate buffer pH = 2 was used to optimize the chromatographic separation of PCC from its degradation products to ensure adequate characteristics, such as resolution and a short time of analysis. Among the various contents of acetonitrile (20%–70%), a 50% content was finally chosen for the determination of PCC and a 30% content of acetonitrile for purity assay and the kinetic analysis of degradation products. The presence of acetonitrile in the mobile phase showed sharp symmetrical peaks of PCC. The presence of phosphate buffer in the chromatographic solvent allowed a distinct separation of PCC. The retention time was not longer than ca. 2.6 min for internal standard and ca. 5.0 min for in mobile phase A or not longer than 5 min, ca. 8.0 min and 15.0 min in mobile phase B. To establish the intermediate precision, another analyst prepared and determined PCC in three solutions of different concentrations. The RSDs ≤1.4% are satisfactory. The detection limit depends on two parameters, such as the composition of the mobile phase and the detection mode, in this case UV detection. In this study the detection limit for PCC was approximately 0.53 µg/ml and its limit of quantification (LOQ) was 1.60 mg/ml.

**Table 1:** MTT cell proliferation assay for 24, 48 and 72 h on normal and cancer cells.

Time (h)	SNU-475	SNU-423	THLE-3
IC_50_ (µg/ml) of PCC			
24	6.98 ± 0.11	7.76 ± 0.45	48.63 ± 0.12
48	6.52 ± 0.23	7.42 ± 0.13	48.52 ± 0.24
72	6.12 ± 0.19	7.21 ± 0.25	48.39 ± 0.43
IC_50_ (µg/ml) of 5-fluoruracil (5-FU)			
24	1.14±0.02 µM	1.25 ± 0.06	1.37 ± 0.15

### Cytotoxic effect of PCC on proliferation of cancer cells

The anti-cancer effect of PCC (Fig. 1) was evaluated on human liver cancer cells SNU-475, SNU-423 and the human liver cell line, THLE-3, by triplicate MTT assays. IC_50_ values for the compound and standard on cell lines tested in this study are shown in Table 1. PCC displayed a high inhibitory effect towards both cancer cells after 24 h. The IC_50_ of PCC was 6.98 ± 0.11 µg/ml and 7.76 ± 0.45 µg/ml against SNU-475 and SNU-423, respectively, as compared with the standard (1.14 ± 0.02 µg/ml), while the IC_50_ for PCC in normal cells was calculated as 48.63 ± 0.12 µg/ml.

**Figure 1:** Chemical structure of PCC.

### PCC induced G1 cell cycle arrest

Development of cancer is due to dysfunction in the regulation of the cell cycle that appears in over-proliferation of cells, although; cancer progression can be strongly limited by conquest of the cell cycle. Hence, the effect of 6.25 µg/ml PCC on cell cycle arrest was investigated. The BrdU and phosphor-histone H3 staining of SNU-475 and SNU-423 cells treated with PCC showed that cell cycle arrest at the S/M phases did not occur (Fig. 2). However, cellular arrest in the G1 phase was detected by using flowcytometery (Fig. 3).

**Figure 2:** PCC arrests the cell cycle in the S/M phase. Cells were incubated with DMSO (control negative) and PCC (6.25 µg/ml) for 24 h with following collection and staining with BrdU and Phopho-Histone H3. Treatment with PCC revealed no significant changes in the BrdU and Phosho-Histone H3 fluorescence intensity which suggests that the cells have not been arrested at S/M phase.

**Figure 3:** Effect of PCC on development of cell cycle using flow cytometry. Momentous cell cycle arrest was identified at G1 phase after 24 and 48 h incubation of the cells with PCC. All data were expressed as the means ± standard error of triplicate measurements. ^∗^*P* < 0.05 compared with the no-treatment group.

### PCC enhanced cytochrome c release and membrane permeability but reduced mitochondrial membrane potential

Because of cytotoxic effect of PCC on SNU-475 and SNU-423 cells, permeability of the membrane was higher than in the control suggesting sustained apoptotic activity in these cells (Figs. 4A and 4B). Loss of mitochondrial membrane potential (MMP) was evidenced as a conceivable mechanism for cell death using MMP dye. The cytoplasm of control cells was stained more intensely than the cells treated with PCC (Fig. 4A). Both SNU-475 and SNU-423 cells treated with PCC for 24 h exhibited a dose-dependent reduction of MMP fluorescence intensity, as a result of collapsed MMP (Figs. 4A and 4B). The fluorescence intensity in the cytosol of SNU-475 and SNU-423 cells treated with PCC was less than control cells suggesting the release of mitochondrial cytochrome c (Fig. 4B).

**Figure 4:** Immunofluorescence study of the effect of PCC. (A) After treatment of the cells with PCC (6.25 µg/ml), Hoechst 33342, cytochrome c, membrane permeability and mitochondrial membrane potential dyes were applied. (B) Representative bar charts indicate a dose-dependent reduction of MMP, elevated cell permeability and cytochrome c release in treated cells. All data were expressed as the means ± standard error of triplicate measurements. ^∗^*P* < 0.05 compared with the no-treatment group.

### PCC induced cytoskeletal rearrangement and nuclear fragmentation

SNU-475 and SNU-423 cells treated with PCC were examined for cytoskeletal and nuclear morphological alteration by phalloidin and Hoechst 33342 staining, respectively. F-actin was stained at the peripheral membrane evidencing the cell shrinkage (Fig. 5). However, nuclear fragmentation and condensation were evident at the concentrations of 6.25 and 3.12 µg/ml of PCC in 24 h but it was more effective at concentration of 6.25 µg/ml (Fig. 6). Additionally, apoptotic chromatin changes increased nuclear intensity suggesting induction of apoptosis by PCC in these cells.

**Figure 5:** Cytoskeletal rearrangement potential of PCC. Cells were treated with various concentration of PCC for 24 h with following fixation and staining with Hoechst 33342 and phalloidin. Dose dependent increase of phalloidin intensity was observed in both WiDr and HT-29 cells. Bar charts are showing the average fluorescence intensity of phalloidin. All data were expressed as the means ± standard error of triplicate measurements. ^∗^*P* < 0.05 compared with the no-treatment group.

**Figure 6:** Nuclear DNA fragmentation occurs by PCC treatment. Cells were treated with PCC (6.25 and 3.12 µg/ml) for 24 h which followed by fixation and staining using Hoechst 33342. DNA fragmentation is indicated by arrows.

### PCC induced membrane blebbing and nuclear condensation

After 24 h treatment of SNU-475, and SNU-423 cells with 6.25 µg/ml of PCC, the apoptotic features were analysed by using fluorescence microscopy. Normal nuclear structure in control cells was displayed as green fluorescence, whereas bright green fluorescence was shown in early apoptotic cells, caused by interposition of acridine orange with the fragmented DNA. Nuclear chromatin pucker and membrane zeiosis, as moderate apoptotic features, were detected after 24 and 48 h. Binding of propidium iodine to denatured DNA was identified by reddish-orange colour after 72 h indicating the late stage of apoptosis (Fig. 7).

**Figure 7:** AO/PI double-staining. Early apoptotic features such as chromatin condensation and blebbing were witnessed after 24 and 48 h of PCC (6.25 µg/ml) treatment. However, after 72 h of PCC treatment (6.25 µg/ml), late apoptosis event was observed. (A) Blebbing of cell membrane after 48 h post-treatment. (B) Late apoptosis after 72 h post-treatment. (C) Chromatin condensation after 48 h post-treatment. (D) Viable cells after 72 h post-treatment.

### PCC enhanced reactive oxygen species production

Following treatment of SNU-475, and SNU-423 cells by PCC for 24 h, ROS production was detected by staining the live cells with DHE. Following rapid oxidation of DHE and production of DCF by ROS, the fluorescence intensity in the cells was quantified by Radiance 2100 confocal microscope (Bio-Rad, Hercules, CA, USA). The cellular DCF fluorescence level was increased almost 1.6 fold in both treated cancer cell lines in compare to control and showed that ROS production can reduce the number of PCC-treated cancer cells in compare to stained untreated normal cells (Fig. 8).

**Figure 8:** Production of ROS based on the effect of PCC (6.25*μ* g/ml). Formation of ROS was significantly increased in both cancer cell lines. All data were expressed as the means ± standard error of triplicate measurements. ^∗^*P* < 0.05 compared with the no-treatment group.

### PCC induced release of lactate dehydrogenase

Lactate dehydrogenase (LDH) is a cytosolic enzyme and serves as a biomarker for cellular cytotoxicity, loss of membrane integrity and cytolysis. PCC significantly induced release of this enzyme at a concentration of 6.25 µg/ml after 24 h showing the potential cytotoxic effect of PCC on SNU-475 and SNU-423 cancer cell lines (Fig. 9).

**Figure 9:** Cytotoxic evaluation of PCC using lactate dehydrogenase (LDH) assay. Bar charts represent that PCC was significantly able to elevate the release of LDH at the concentration of (6.25 µg/ml). All data were expressed as the means ± standard error of triplicate measurements. ^∗^*P* < 0.05 compared with the no-treatment group.

### PCC mediated NF-*κ*B translocation

A substantial suppressive effect against TNF-*α*-stimulated translocation of NF-*κ*B in the SNU-475 and SNU-423 cells was identified at a PCC concentration of 6.25 µg/ml (Fig. 10). Non-stimulated states distinguished by the high NF-*κ*B fluorescence intensity in the cytoplasm of normal cells. High fluorescence intensity was observed in the nucleus of cancer cells. PCC stimulates apoptosis in these cells by activating TNF-*α* which translocates NF-*κ*B and gradually reduces the fluorescence intensity in the cytoplasm.

**Figure 10:** Translocation of NF-*κ*B. After treatment of both cancer cells by several concentration of PCC for duration of 3 h, the cells were exposed for 30 min to TNF-*α* (1 ng/ml). Results disclosed no significant cytoplasmic to nucleus translocation of NF-kB. All data were expressed as the means ± standard error of triplicate measurements. ^∗^*P* < 0.05 compared with the no-treatment group.

### PCC upregulated expression of glutathione reductase

Real time profiler qPCR-array was used to identify the expression of the genes involved in the cellular stress response in PCC-treated SNU-475 an SNU-423 cells. In this method, 84 human genes involved in oxidative stress and antioxidant defence, the antioxidant peroxiredoxin (PRDX) family and redox control were examined. Results showed that the antioxidant related and oxidative stress genes were differently expressed in the cells in response to PCC. Interestingly, glutathione reductase was noticeably up-regulated by more than 80 fold in SNU-423 and more than 100 fold in SNU-475 as compared with normal cells (*P* < 0.05). These findings were validated by qPCR (Figs. S1 and S2).

### PCC induced caspase 3/7, 8 and 9

The bioluminescent intensity of caspase 3/7, 8 and 9 activities of cancer and normal cells was measured at 6, 12, 18, 24, 30, 36 and 42 h time points after PCC treatment. A significant increase of caspase 3/7, 8 and 9 activities was detected after 18 and 24 h of PCC exposure in the cancer cells (Fig. 11). The maximum activity of caspase 9 was observed in both PCC-treated cancer cell lines after 18 h (4.8 fold for SNU-423 and 5.0 fold for SNU-475), whereas after 24 h of PCC exposure, the caspase 3/7 and 8 activities were increased to a peak in both cancer cells and then gradually decreased at the later time points. This finding suggests that PCC can induce apoptosis in the liver cancer cells through activation of caspase 9 and 8. In addition, the activity of caspase 3/7, 8 and 9 were inhibited by the caspase inhibitor, Z-VAD-FMK (10 µM), in the presence of PCC (6.25 µg/ml) (Table S1).

**Figure 11:** Time-dependent activation of caspase 3/7, 8 and 9 by PCC (6.25 *μ* g/ml). The results disclosed a significant activation in caspase 3/7, 8 and 9 in a time-dependent manner. All data were expressed as the means ± standard error of triplicate measurements. ^∗^*P* < 0.05 compared with the no-treatment group.

### PCC induced both mitochondrial and extrinsic pathways

Western blot analysis disclosed a reduction in the expression level of Bcl-2 (26KDa) and Bcl-xL (30KDa) in PCC treated SNU-475 and SNU-423 cells. In both liver cancer cell lines, the level of Bcl-2 an Bcl-xL were substantially altered at 6.25 µg/ml PCC with further down-regulation observed at 12.5 and 25 µg/ml (Fig. 12). In addition, upregulation of p53 (53KDa) and Bax (23KDa), cleavage of Bid (22KDa) to its truncated form (15kDa) as well as cleavage of caspase-7 (20KDa), 8(43KDa), and 9(37KDa) were evident in both cancer cell lines (Fig. 12). Cleavage of caspase 3 subunits including the 17 and 11 kDa subunits, was identified in PCC-treated cancer cells, whereas, cleavage was not detected in normal cells with a similar dosage of treatment. This finding suggests that PCC induces apoptosis through both mitochondrial and extrinsic pathways. PCC also modulates binding of truncated Bid to Bax resulting in the release of cytochrome c from mitochondria.

**Figure 12:** Western blot analysis of cancer and normal cell lines. Cells were treated with 3.12 and 6.25 µg/ml of PCC for 24 h. Proteins were transferred to a membrane and followed by probing with antibodies. Normalization of band densities of treated samples were accomplished based on the control. The results represent significant increase in the expression level of caspase 3, 7, 8, 9, p53, Bax and conversion of Bid to its truncated form (tBid), whereas decrease in Bcl-2 and Bcl-xL level.

### Annexin-V-FITC assay

Cells were pre-treated with cell membrane permeable calcium chelator EGTA/AM (25 µM) for 1 h followed by addition of complex (6.25 µg/ml) for 24 h. Both cancer cell lines (SNU-475 and 423) were stained with Annexin V FITC and PI then subjected to flow cytometry analysis. Our data indicated that calcium depletion did not inhibit complex-induced apoptosis (Fig. 13).

**Figure 13:** Quality assay of apoptosis. Cells were treated with EGTA/AM (25 µM) prior to exposure to PCC 6.25 µg/ml. Apoptosis analysis shows (A and D): the untreated cells as the control; (B and E): 24 h PCC-treatment of the cells; (C and F): 24 h PCC-treatment+ EGTA/AM.

## Discussion

The ability of malignant cells to evade apoptosis is a hallmark of cancer. Thus, a comprehensive perception of apoptotic signaling pathways is mandatory for discovery of target selective therapeutic drugs. Through investigation of the properties of PCC as a new derivative of piperazine in the current study, we found that this agent is potentially cytotoxic against liver cancer cells. In particular, PCC can simultaneously induce both extrinsic and intrinsic apoptotic signaling pathways in these cells. By calculating the mean IC50 THLE-3/mean IC50 of SNU-475 or SNU-423 we showed that PCC selectivity is much higher for cancer rather than normal cells which confirm its potential as a good candidate as anti-cancer agent. This feature can be considered as a prominent property of this compound in cancer cell treatment. Our findings provide molecular evidence for potential cytotoxic properties of PCC in the liver cancer cells by its stimulation of both extrinsic and intrinsic apoptotic-dependent signaling pathways.

Apoptosis consists of morphological and biochemical changes. Following a death signal, morphological events initiated by cell shrinkage and chromatin condensation proceed to membrane blebbing and nuclear fragmentation and finally end with apoptotic body formation (Elmore, 2007). To address whether PCC induces cytological alterations in the liver cancer cell lines, we monitored the cell membrane, LDH and cytochrome c release, ROS production, mitochondrial membrane potential, cytoskeleton, nuclear fragmentation and NF-*κ*B translocation in PCC treated cells. Results showed that PCC can stimulate cytoskeletal shrinkage-related reorganization. This compound substantially damages membrane integrity at a concentration of 6.25 µg/ml, leading to LDH release from the cells as a marker of cytotoxicity (Fig. 9). Analysis of membrane blebbing and chromatin condensation by using AO/PI staining revealed the morphological changes relevant to the apoptotic event (Figs. 6 and 7) (Aarts et al., 2012). By increasing the period of the cell exposure to PCC from 24 to 72 h, modifications of the early to the late stage of apoptotic events appeared, suggesting that a prolonged treatment of cancer cells with PCC can activate necrosis in these cells (Gasparri, Cappella & Galvani, 2006; Tentner et al., 2012; Wang et al., 2012). Cell cycle distribution was furthered investigated to support the occurrence of apoptosis in the cancer cells through BrdU and Phospho-Histone H3 staining (Gasparri, Cappella & Galvani, 2006; Wang et al., 2012). However, neither BrdU attachment nor H3 staining in the mitotic stage was identified, indicating that there was no significant difference in the number of cells in the S/M phases. Based on flow cytometric analysis, the cells were observed to be arrested at the G1 or G2 phases. This finding confirms that cell death is triggered by apoptosis (Liu et al., 2012; See et al., 2010). Mitochondria are the main source of ROS which regulate survival or death of cells. Our data show an extensive enhancement in the ROS levels in the PCC (6.25 µg/ml) treated cells. The enzyme, GR, as an oxidative stress indicator, plays an important role in the suppression of reactive oxygen species and in anti-oxidant function. Enhanced ROS production is known to stimulate *de novo* synthesis of GR (Wu et al., 2004). In our study, we assume that PCC stimulates ROS production through upregulation of GR (Figs. S1 and S2).

Disproportionate ROS production diminishes mitochondrial membrane potential leading to cytochrome c release from mitochondria into the cytoplasm. An increased mitochondrial cytochrome c level in the cytoplasm is a key initiative signal for induction of the intrinsic apoptosis pathway by PCC (Fig. 4) (Elmore, 2007; Ling, Lin & Perez-Soler, 2008). Thus, PCC can be seen as a potential inducer of morphological modifications downstream of apoptotic molecular events in the liver cancer cells associated with its cytotoxic potential.

Apoptosis is specified by a series of morphological modifications which are triggered by various molecular events to stimulate cells to undergo cell death rather than recovery. Yet, there are little data showing that the piperazine compounds can induce apoptosis pathways associated with their cytotoxic properties. Recent studies have demonstrated the cytotoxic effect of some piperazines derivatives such as *β*-elemene piperazine, 1,4-bis-(4-(1H-benzo[d]imidazol-2-yl-phenyl) piperazine, and chloroalkyl piperazine and 6-(4-substituted piperazine-1-yl)-9-(*β*-D-ribofuranosyl) purine in cancer cells. However, only the extrinsic pathway of apoptosis is activated by these compounds (Baumgartner et al., 2007; Guo, Tong & Li, 2004; Sampson III et al., 2011; Tuncbilek et al., 2012; Yu et al., 2011). To further support the role of PCC as a novel piperazine derivative with pro-apoptotic properties, we analyzed the apoptotic pathways in the liver cancer cell lines. Results showed that PCC enhanced the release of mitochondrial cytochrome c which activates caspase 9 by 4.8–5.0 folds in both liver cancer cells (Baliga & Kumar, 2003). Interestingly, activated caspase-8 is also increased by about 5-fold in both cancer cells, suggesting that PCC-induced apoptosis is mediated by more than one pathway. Following cell excitation, calcium ions are released from mitochondria to regulate several cellular processes such as apoptosis. Therefore, prolonged elevation of cytosolic calcium ions causes cell death (Rizzuto et al., 2008). In addition, mitochondrial calcium ion uptake alters the mitochondrial permeability which switches on apoptotic events in response to the stress. Increase of calcium ion levels occurs at both the early and late stages of apoptosis (Rizzuto et al., 2008). Hence, intracellular calcium ion elevation causes cell death through apoptosis pathways (Kruman, Guo & Mattson, 1998; Lynch et al., 2000; Tombal, Denmeade & Isaacs, 1999). On the basis of the absence of cytosolic free calcium evaluated by using a calcium chelator (EGTA/AM) and flow cytometry analysis of Annexin-V in the PCC treated cells, an increase in the number of cells was detected. Therefore, caspase 8 has been activated by PCC independent of intracellular calcium concentrations.

In liver cancer, development of resistance against various therapeutic interventions, such as chemotherapy, is linked to the expression of Bcl-2 and Bcl-xL (Friesen et al., 1996; Hyer et al., 2008; Wieder et al., 2001). Bcl-2 is an anti-apoptotic mediator that is expressed in different cancer types and serves as a checkpoint in execution of the caspase cascade and mitochondrial dysfunction (Elmore, 2007; Ling, Lin & Perez-Soler, 2008; Park et al., 2013). In addition, Bcl-xL blocks cell death through regulation of mitochondrial homeostasis (Baliga & Kumar, 2003; Elmore, 2007). Furthermore, the tumor suppressor P53 is an apoptosis mediator in numerous cells activated by DNA damage which triggers apoptosis to eliminate permanently damaged cells (Chou et al., 2010). Dysfunction or down-regulation of p53 can induce tumor progression and resistance to chemotherapy (Gerasimenko et al., 2002). Our experimental data show that PCC reduces the levels of Bcl-2 and Bcl-xL, but increases p53 concentration in the PCC- treated liver cancer cells. Cytotoxic drugs can mediate cleavage of Bid through activation of caspase 8 (Friesen et al., 1996; Hyer et al., 2008). In the absence of interaction between ligand and death domain adaptor protein, some drugs may activate caspase-8 (Wieder et al., 2001). Following the conversion of Bid to its truncated form (tBid), mitochondrial cytochrome c is released into the cytoplasm to activate Bax (Schug et al., 2011). In this study, the process of cell death was associated with upregulation of Bax and caspase-8/Bid pathway in PCC treated cells (Hajrezaie et al., 2014; Lee et al., 2012). In addition, we showed that anticancer potential of PCC can be mediated by reduction in the activation of NF-*κ*B signaling pathways. Targeting NF-*κ*B signaling pathway by drugs has been considered as novel chemotherapeutic objectives in cancer therapy (Elmore, 2007; Shakibaei et al., 2013; Su et al., 2013). Evidence showed a linkage between anticancer drug resistance and enhanced activity of the NF-*κ*B pathway (Su et al., 2013). NF-*κ*B antagonists inhibit binding of this molecule to DNA resulting in suppression of cell proliferation.

## Conclusion

Evaluating the cytotoxic properties of PCC in the current study suggests that this compound has potential as an anticancer agent against liver cancer cells. PCC simultaneously induces both internal and external apoptosis pathways, and hence, can be nominated as a potential anti-cancer agent for future *in vivo* studies.

## Supplemental Information

10.7717/peerj.1588/supp-1 Supplemental Information 1 Caspase activity

10.7717/peerj.1588/supp-2 Supplemental Information 2 actin1

10.7717/peerj.1588/supp-3 Supplemental Information 3 actin 2

10.7717/peerj.1588/supp-4 Supplemental Information 4 ldh1

10.7717/peerj.1588/supp-5 Supplemental Information 5 ldh

10.7717/peerj.1588/supp-6 Supplemental Information 6 caspase

10.7717/peerj.1588/supp-7 Supplemental Information 7 dhe

10.7717/peerj.1588/supp-8 Supplemental Information 8 cyt1

10.7717/peerj.1588/supp-9 Supplemental Information 9 cyt 2

10.7717/peerj.1588/supp-10 Supplemental Information 10 dhe 2

10.7717/peerj.1588/supp-11 Supplemental Information 10 permeability

10.7717/peerj.1588/supp-12 Supplemental Information 12 caspase 2

10.7717/peerj.1588/supp-13 Supplemental Information 13 nfkb

10.7717/peerj.1588/supp-14 Supplemental Information 14 nfkb2

10.7717/peerj.1588/supp-15 Supplemental Information 15 permiability

10.7717/peerj.1588/supp-16 Supplemental Information 16 mmp1

10.7717/peerj.1588/supp-17 Supplemental Information 17 mmp2

10.7717/peerj.1588/supp-18 Supplemental Information 18 Human oxidative stress and antioxidant defence qPCR-array was used to identify genes significantly up- or down-regulated in PCC treated cancer cells. Gene profiling analyses were performed three times in independent experiments. (Arrow indicates location of GR in the scatterplots).

## Additional Information and Declarations

### Data Availability

The following information was supplied regarding data availability: The raw data is supplied as Supplemental Information.
